# Deciphering the binding mechanism of an anti-cancer phytochemical plumbagin with calf thymus DNA using biophysical and *in silico* techniques

**DOI:** 10.3389/fchem.2023.1248458

**Published:** 2023-08-29

**Authors:** Abdul Rahaman, Farah Anjum, Aknita Kumari, Alaa Shafie, Mahafooj Alee, Omnia Badr, Shaheer Hasan Khan, Amal Adnan Ashour, Ali Hazazi, Sultan Arif, Xin-An Zeng

**Affiliations:** ^1^ Guangdong Key Laboratory of Food Intelligent Manufacturing, Foshan University, Foshan, Guangdong, China; ^2^ School of Food Science and Engineering, Foshan University, Foshan, China; ^3^ Department of Clinical Laboratory Sciences, College of Applied Medical Sciences, Taif University, Taif, Saudi Arabia; ^4^ School of Food Science and Engineering, South China University of Technology, Guangzhou, China; ^5^ Department of Genetics and Genetic Engineering, Faculty of Agriculture, Benha University, Qalyubia, Egypt; ^6^ Enzymology and Nanotechnology Laboratory, Interdisciplinary Biotechnology Unit, Aligarh Muslim University, Aligarh, India; ^7^ Department of Oral and Maxillofacial Surgery and Diagnostic Sciences, Faculty of Dentistry, Taif University, Taif, Saudi Arabia; ^8^ Department of Pathology and Laboratory Medicine, Security Forces Hospital Program, Riyadh, Saudi Arabia; ^9^ Department of Plastic Surgery and Burn Unit, Security Forces Hospital, Riyadh, Saudi Arabia; ^10^ Overseas Expertise Introduction Centre for Discipline Innovation of Food Nutrition and Human Health (111 Centre), Guangzhou, China

**Keywords:** cancer, Plumbagin, groove binder, biophysical, circular dichroism, molecular simulation

## Abstract

Plumbagin (PLM), a plant derivative, is well known for a wide range of therapeutic effects in humans including anti-cancer, anti-inflammatory, anti-oxidant, and anti-microbial. Cytotoxic and genotoxic potential of this phytochemical has been studied which demands further insight. DNA being a major target for several drugs was taken to study against PLM to understand its effects on the cellular system. UV-Vis spectroscopy has indicated the binding of PLM to ctDNA and dye displacement assays have confirmed the formation of PLM-ctDNA complex. The insignificant changes in circular dichroism spectra suggested that PLM is not affecting the structural makeup of the ctDNA, hence the binding could be peripheral and not intercalating. Further, the relative viscosity and minimal change in melting temperature upon the complex formation supported this finding and confirmed the groove binding of PLM. Molecular docking analysis and simulation studies also show PLM as a minor groove binder to DNA and provide details on the interaction dynamics of PLM-DNA complex. Docking followed by a 100 ns simulation reveals the negative Gibbs free energy change (∆G = −6.6 kcal mol^−1^), and the formation of a stable complex. The PLM- DNA complex with stable dynamics was further supported by different parameters including RMSD, RMSF, SASA, Rg, and the energy profile of interaction. This study provides an insight into the cytotoxic and genotoxic mechanism of PLM which can be a crucial step forward to exploit its therapeutic potential against several diseases including cancer.

## 1 Introduction

Plumbagin (PLM) [5- hydroxy-2-methyl-1,4-naphthoquinone] is an established anti-cancer agent, the effects of which have been studied in breast cancer, ovarian cancer, lung cancer, acute promyelocytic leukemia, and prostate cancer (Aziz et al., 2008; Manu et al., 2011; Subramaniya et al., 2011; Lai et al., 2012; Sinha et al., 2013; Niu et al., 2015; Liu et al., 2017). PLM is a plant derivative of Plumbago zeylanica and belongs to one of the largest and most diverse groups of plant metabolites (Chen et al., 2009). In cancer cells, PLM has been critical in inhibiting growth, invasion, and metastasis; induction of apoptosis; and anti-angiogenesis. PLM causes the suppression of major signalling molecules which are essential for cancer cell development including AKT/mTOR, nuclear factor-kappa B, and signal transducer and activator of transcription 3 (Aziz et al., 2008; Manu et al., 2011; Sinha et al., 2013).

Deoxyribonucleic acid (DNA) is the prime site for the storage of genetic information in humans. If this information gets compromised at any level, the results can be dangerous and deadly, because DNA has its role in multiple life processes including replication, transcription, gene expression, etc. (Li et al., 2012). DNA-small molecule interaction has gained much interest in the fields of biological and chemical sciences which demands to acquire an in-depth understanding of its mechanism (Lefstin and Yamamoto, 1998; Rajendiran et al., 2008; Rehman et al., 2015). These types of interactions provide further insights into the structural properties of DNA with the mode of binding and mechanism of the small molecules influencing DNA functioning and their consequences.

DNA can bind to small molecules or drugs through covalent or non-covalent interactions, the dominant ones being the non-covalent bonds, which are further classified into intercalations, electrostatic interactions, and groove binding interactions (Sarkar et al., 2008). The complexity of these interactions always demands an in-depth investigation to fully exploit their potential (Froehlich et al., 2011). Hence, there is always a scope for improvement to better understand the significance and impact of the binding of a particular compound with DNA.

In the present study, calf thymus DNA (ctDNA) was interacted with PLM. Different spectroscopic, thermal stability and hydrodynamics experiments were performed to study the interaction, helix melting, and viscosity of DNA in the presence of PLM. Molecular docking and simulation studies were performed to establish the mode of binding and understand the dynamics of PLM-DNA complex. All the results provided important insight regarding PLM-ctDNA complex formation and the mechanism of PLM action while interacting with DNA. While providing an important step towards studying the PLM mechanism inside the cell, this work will further require a rigorous clinical research to establish the discussed finding and impact.

## 2 Materials and methods

### 2.1 Materials

PLM, ctDNA, ethidium bromide (EB), acridine orange (AO), and Hoechst 33,258 were procured from Sigma Aldrich (USA). Sodium phosphate buffer (20 mM; pH 7.4) was used as the solvent for most of the experiments.

### 2.2 UV-vis spectroscopic analysis

The absorption spectra were recorded using a UV-1800 Shimadzu spectrophotometer (Japan) in the range 220–320 nm for PLM and PLM-ctDNA complex. The baseline was corrected with the buffer (sodium phosphate, pH 7.4; 25°C) and the concentration of PLM was fixed at 20 µM, while the concentration of ctDNA varied from 2 to 20 µM.

### 2.3 Dye displacement measurements

The fluorescence spectra of the samples were obtained using a Shimadzu RF-5301pc spectrofluorometer (Japan). In the EB displacement assay, the concentration of EB (20 µM) was kept fixed with ctDNA (40 µM), while the concentration of PLM was varied between 5–50 µM. The emission spectra of the EB-ctDNA complex were recorded between 520–670 nm, keeping excitation fixed at 360 nm. In the AO displacement assay, the emission spectra of the AO-ctDNA complex were recorded within the range of 490–630 nm, with a fixed excitation wavelength at 480 nm. The slits for both excitation and emission spectra were set at 10 nm. The concentration of DNA was fixed at 40 µM while the concentration of PLM was varied between 5–50 µM for titration. Similarly, the DNA-Hoechst 33,258 complex spectra were obtained after excitation at 343 nm, and the emission spectra in this experiment were recorded between 350–600 nm. The Stern–Volmer for all three displacement experiments was plotted based on fluorescence quenching to predict the binding site of PLM while forming the complex.

### 2.4 Circular dichroism (CD) measurements

CD spectra of ctDNA and PLM-ctDNA complex were measured using a JASCO-J-813 spectropolarimeter with a Peltier-type temperature controller. The spectra were recorded at 298 K from 220 to 300 nm, using a quartz cell with a path length of 0.1 cm. The molar ratios of the PLM-ctDNA complex were 1:0, 1:1, and 1:2. The CD spectra were expressed in CD (mdeg) units after subtraction of corresponding blanks.

### 2.5 Viscosity measurements

To further understand the binding mechanism between PLM and ctDNA, viscosity measurements were performed. The experiment was carried out at a constant temperature of 25°C ± 0.5°C using a UBBELOHDE viscometer. The concentration of ctDNA was kept constant at 150 µM, while different concentrations of PLM were used. The flow time was measured using a digital stopwatch, and the mean of three replicates was recorded for each sample. The relative specific viscosity (η/ηO)1/3 values were determined and plotted against the ratio of [ligand]/[DNA] concentrations. Here, ηO and η represent the viscosity contributions of DNA in the absence and presence of PLM, respectively.

### 2.6 Helix melting studies

UV-spectrophotometer (UV-1800 Shimadzu, Japan) using 1 × 1 cm quartz cuvettes, coupled with a thermostat bath was utilized to conduct the helix melting studies. The analysis of ctDNA double-stranded structure was done in the presence and absence of PLM at 260 nm, with temperature variation. All melts were performed using quartz cells with a 1 cm path length. The temperature was varied from 35°C to 90°C, and the relative absorbance was plotted against the temperature. The DNA melting temperature (Tm) was calculated as the midpoint of the transition observed in the plot.

### 2.7 Molecular docking analysis

AutoDock Vina was used to study the interaction between PLM and ctDNA. The ctDNA molecule used for docking studies was the dodecamer d (CGCGAATTCGCG)2 (PDB ID: 1BNA), and its 3D structure was obtained from the Protein Data Bank. Prior to docking, MGL-Tools-1.5.6 was used to add polar hydrogen atoms and Gasteiger charges to the ctDNA molecule. A grid box of dimensions 58 × 72 × 112 Å was set up, with the center of the grid located at X = 14.759, Y = 20.984, and Z = 8.812, and a spacing of 1 Å was used to cover the entire DNA molecule. The structure of PLM, obtained from PubChem (CID: 10,205) in sdf format, was converted to pdb format using Chimera-1.10.2 and optimized using Avogadro software. The docking calculations were performed using AutoDock vina with an exhaustiveness of 100, and the Broyden-Fletcher-Goldfarb-Shanno algorithm was used. The PyMOL software package was used to analyze the output and present the data in 3D form. LigPlot+ (version v.2.2.8) was used to plot the 2D representation of the interacting residues with the ligand molecule (Wallace et al., 1995).

### 2.8 Molecular dynamics simulation

The study of the complex formed by PLM with DNA was carried out using molecular dynamics simulations (MDS) with GROMACS 2018.1 (Páll et al., 2015). The amber99sb- ILDN force field was used to simulate the system, and the structures were solvated in a triclinic box using the TIP3P water model. To neutralize the structures, 22 sodium ions were added. The ligand topology was generated using the antechamber program in AmberTools19, which is a software suite for carrying out MDS. The energy minimization step was performed to remove any weak Van der Waals contacts and optimize the structures of both the DNA and PLM-DNA complex. This was done using the steepest descent algorithm with 5,000 steps. After the energy minimization step, both systems were equilibrated for NVT using the V- rescale thermostat for 100 ps at a temperature of 300 K. The NPT ensemble was then used to further equilibrate the systems for 1,000 ps at a pressure of 1.0 bar using the Parrinello-Rahman barostat. The Particle-Mesh Ewald method is a widely used algorithm in MDS for computing long-range electrostatic interactions. It combines real space and reciprocal space calculations to calculate the electrostatic interactions between charged particles. The Van der Waals interactions were set at 1.2 nm, which is a typical value used in many MDS. The Linear Constraint Solver (LINCS) algorithm is used to constrain covalent bond lengths and bond angles during MDS. This algorithm is used to maintain the geometry of the molecule during the simulation and prevent unrealistic bond lengths or angles from occurring. The LINCS algorithm is especially useful in simulations that involve stiff molecules such as proteins or nucleic acids. The heavy atom-H bonds were also constrained using this algorithm to prevent unrealistic movements of the atoms during the simulation. The gmxrms, gmxrmsf, gmxgyrate, gmxhbond, gmx sasa utilities were used to calculate root mean squared deviation (RMSD), root mean squared fluctuation (RMSF), radius of gyration (Rg), hydrogen bonds, and solvent accessible surface area (SASA), respectively. The MM-PBSA calculations were performed after simulation to calculate the binding energy of ligands and receptors (Kumari et al., 2014).

## 3 Results and discussion

### 3.1 UV–vis spectroscopy

UV-Vis spectroscopy is a prevalent technique for investigating the interaction of small molecules, drugs, and biological molecules such as proteins or DNA (Shi et al., 2015; Ahmad and Ahmad, 2018). In this study, UV-Vis spectroscopy was employed to analyze the absorbance spectra of the PLM-DNA complex. The absorbance of PLM alone was observed at 270 nm as its characteristic peak, but when DNA was added, there was a significant increase in absorption with a shift in the position of the peak **(** Figure 1 **)**. The decreased absorbance (hypochromicity) and red-shift in the maxima suggest an intercalative mode of binding between DNA and small molecules, according to previous studies (Rahban et al., 2010). However, our findings, combined with the existing literature, led us to suggest that PLM may interact with ctDNA through a non-intercalative mode (Wang et al., 2002; Shahabadi and Hadidi, 2012). While this technique does not provide detailed mechanistic insights into the possible binding mode of PLM-ctDNA, it served as a basis for further experiments to establish these results.

**FIGURE 1:** UV spectra of PLM with and without ctDNA.

### 3.2 Competitive displacement assay

The common fluorophores were used to study the binding mode of PLM-ctDNA interaction. EB is a strong intercalative agent; its fluorescence intensity increases in the presence of DNA (Song et al., 2000). Researchers have found out that the enhanced emission intensity of EB-DNA complex can be quenched by the addition of another molecule if this molecule also binds through the same mode as EB. While binding to the similar position the molecule can displace the EB and this results in the decreased fluorescence intensity of the EB–DNA complex (Wu et al., 2011; Li et al., 2014). Acridine orange dye (AO), behaves the same way as, i.e., intercalation as in EB (Sayed et al., 2016). The result suggests that PLM does not have a significant effect on the binding of EB and AO to ctDNA. Therefore, the lack of change in fluorescence upon the addition of PLM suggests that PLM does not interfere with the intercalation of EB and AO into ctDNA (Figure 2A). This led us to the conclusion that PLM was not able to replace EB or AO while forming the complex with ctDNA, suggesting that PLM does not bind through intercalative binding mode. Hoechst 33,258 is a known minor groove binder that was used to further elucidate the binding of PLM with ctDNA (Kakkar and Garg, 2002; Guan et al., 2006). There was a significant decrease in the fluorescence spectra of Hoechst-ctDNA complex upon the addition of PLM to the said complex, suggesting PLM binds to DNA through the same mode as Hoechst 33,258 dye (Figure 2B). That is, PLM could replace Hoechst from the grooves of DNA thus decreasing the fluorescence. This quenching of the Hoechst-ctDNA complex upon the addition of PLM provides additional evidence to confirm non-intercalative binding mode of PLM to ctDNA (Figure 2C).

**FIGURE 2:** Dye displacement assays with varying concentrations of PLM; **(A)** Ethidium bromide, **(B)** Acridine orange, **(C)** Hoechst, **(D)** Combined Stern–Volmer for PLM-ctDNA binding constant.

The KSV values of all three displaced dyes (EB, AO and Hoechst) bound to ctDNA by PLM were calculated, using the Stern–Volmer plot (Lakowicz, 2006) as shown in Figure 2D. KSV values of EB, AO and Hoechst were 0.21 × 10^4^ (M^−1^), 4.25 × 10^4^ (M^−1^) and 12.6 × 10^4^ (M^−1^). The results clearly indicate that the KSV value for Hoechst-ctDNA complex was significantly higher than that for EB/AO-ctDNA complex, indicating PLM binding at the position of Hoechst in ctDNA. This suggests that PLM may bind to the DNA in the minor groove, possibly after displacing Hoechst.

### 3.3 Circular dichroism study

CD is a highly informative and sensitive method that helps to comprehend changes in the secondary structure of biological molecules, such as DNA and proteins, when they interact with small molecules (Holm et al., 2010). These modifications depend on the non-covalent interactions between DNA and small molecules and can lead to changes in the intrinsic CD spectral behavior (Zhang et al., 2011). The CD spectrum of ctDNA showed a positive peak at approximately 276 nm, which is attributed to base stacking, and a negative peak at around 245 nm, which is indicative of right-handed double helical DNA helicity (Li et al., 2014), (Figure 3). The intensity and position of these peaks can be significantly altered by the interaction of DNA with small molecules (Ivanov et al., 1973; Uma Maheswari and Palaniandavar, 2004). Studies have indicated that when DNA binds with small molecules through intercalation, it causes significant alterations in base stacking and helicity, while the electrostatic interactions and groove binding have no significant impact on these characteristics of DNA structure (Mergny et al., 1992; Jain et al., 2003). From Figure 3, it is clear that the addition of PLM to ctDNA did not cause any significant perturbations in the CD spectra. These results further suggest that PLM acts as a groove binder for DNA rather than an intercalator.

**FIGURE 3:** Effect of PLM (varying concentrations; 1:1 and 1:2) on CD spectra of ctDNA.

### 3.4 Viscosity measurement

A classical intercalative case of ligand binding increases the length of DNA because of the stacking of small molecules between the base pairs; hence, increasing the viscosity of the DNA (Satyanarayana et al., 1992; 1993). Whereas, when the small molecules bind to DNA through groove binding or electrostatic mode, no significant change in viscosity is found (Shahabadi et al., 2011; Raman et al., 2012). To further confirm the non-intercalative binding mode of PLM to ctDNA, the relative specific viscosity (η/ηO)1/3versus [ligand]/[DNA] ratio was plotted. The results showed an insignificant change in the viscosity upon the continued addition of PLM to ctDNA (Figure 4), which is consistent with groove binding rather than intercalation. These results further concrete the groove binding mode and rule out the possibility of intercalation.

**FIGURE 4:** Effect of PLM binding on the relative viscosity of ctDNA.

### 3.5 Helix melting study

The melting of double-stranded DNA (dsDNA) is referred to as the separation of two strands of the DNA, and the temperature at which half of the DNA is in double-stranded and the other half is in single-stranded form is called the melting temperature (Tm) (Wijeratne et al., 2011). The absorbance intensity of DNA shows a sharp increase as the two strands separate because the extinction coefficient of dsDNA bases at 260 nm is much less as compared to DNA in single-stranded form (Roy et al., 2009; Wang et al., 2012). The intercalative binding mode results in a sharp increase in Tm (4°C–8 °C), whereas groove-binding interaction shows no effect or less effects on Tm (Wilson et al., 1994). In this study, from the DNA melting profiles, the estimated Tm were found to be 66 and 70 for the unbound ctDNA and PLM-bound DNA, respectively (Figure 5). The insignificant increase in Tm upon PLM binding strengthens the earlier experimental claims that PLM binds to ctDNA through groove-binding mode.

**FIGURE 5:** Helix melting profile of ctDNA in absence and presence of PLM.

### 3.6 Molecular docking analysis

Molecular modelling and docking studies were executed for obtaining details about the PLM–DNA interaction; this further validate the *in vitro* experimental results. The 2D and 3D representations of conformations were selected, among the 10 binding modes, based on the lowest binding free energy (−6.6 kcal mol^−1^). The binding constant value for the PLM-DNA complex was calculated to be 6.92 × 10^4^ M^−1^. The molecular docking analysis revealed that PLM formed four hydrogen bonds with the nitrogenous bases along the helix and Van der Waal interactions were observed for minor groove binding (Figure 6). Thus, the molecular docking analysis supports the results obtained from the *in vitro* studies, indicating that PLM binds to the groove of DNA. The further validation of the stability of the complex was analyzed by molecular dynamics simulation.

**FIGURE 6:** Molecular docking analysis of PLM-DNA complex showing **(A)** 3D image of PLM-DNA complex, **(B)** 2D image of PLM showing interaction with DNA, and **(C)** LigPlot of PLM-DNA complex showing hydrogen bonding and Van Der Waal interactions.

### 3.7 Molecular simulation analysis

#### 3.7.1 RMSD

MDS was performed to evaluate the stability of DNA and its complex with PLM over 100 ns. The RMSD values of both systems were calculated relative to their initial structures. It was observed that the RMSD value of DNA reached equilibrium after about 20 ns with a value of around 0.35 nm. The average RMSD of DNA was 0.321 nm and PLM-DNA was 0.253 nm, showing a difference of 0.068 nm in the RMSD due to the formation of complex. The lowered average RMSD value of the PLM-DNA complex indicates its stability in an aqueous environment. The RMSD of the ligand molecule was also calculated and found to be less than 0.05 nm throughout the simulation period, further confirming the stability of the complex. The visual analysis of the trajectories also supports the stability of both the DNA and DNA-PLM complex systems (Figure 7A). These results suggest that the PLM-DNA complex is stable and can withstand fluctuations in the aqueous environment.

**FIGURE 7:** MDS analysis elaborating the interaction dynamics and the stability of the PLM-DNA complex. **(A)** RMSD plot, **(B)** RMSF plot, **(C)** Rg plot, **(D)** SASA plot, **(E)** Potential energy, **(F)** Total energy.

#### 3.7.2 RMSF

The RMSF values of the DNA and its complex with PLM was calculated as a result of averaging all the snapshots during the 100 ns simulation implying the determination of the dynamic behaviour of the residues in DNA. These values provide insight into structural flexibility and fluctuations of different regions. If fluctuations are more, it means that the residues are unstable, otherwise residues are said to be stable. The RMSFs of Cα atoms of the DNA and DNA- PLM complex was shown in Figure 7B. Most of the residues in the DNA and its complex were observed to have values below 0.2 nm except for the terminal residues and the general shape of the fluctuation curve for both complexes was similar. However, the terminal residues also show decreased RMSF values when complexed with PLM conferring to stabilizing the fluctuation of residues as a result of interaction with the ligand molecule.

#### 3.7.3 Compactness and SASA

Rg is known to be a measure of stability in a system during MDS. Biomolecular structures that are compact tend to have less variation in Rg values, while those that are expanded tend to have higher Rg values. The Rg values of both the DNA and DNA-PLM complex were plotted against time in Figure 7C. The results showed that the binding of PLM to the DNA molecule slightly increased the compactness of the structure compared to the free DNA molecule, as evidenced by a slight decrement in the Rg values of the DNA-PLM complex. The Rg values remained relatively constant over the entire simulation time of 100 ns, indicating that the systems were in equilibrium.

The SASA variations of both the systems, DNA and PLM-DNA complex, were shown in Figure 7D. As observed for Rg, the SASA values for both the systems were also found to be approximately much alike which further describes the stability of DNA and DNA-PLM complex.

#### 3.7.4 Energy analysis

The physicochemical parameters of the systems were also analyzed to confirm their stability. The potential energy and total energy of both the DNA and DNA-PLM complex systems were examined, as depicted in Figures 7E, F. The smooth curves observed for both parameters indicate that the systems reached equilibrium and remained stable throughout the 100 ns simulation period.

## 4 Conclusion

PLM is a widely used anti-cancer phytocompound which has several other effects on cellular system. The mechanism of its effects and possible consequences needs to be understood for better utilization of its potential and to minimize its adverse outcomes. This study shows that PLM interacts with DNA to form a stable complex targeting the minor groove of this double-stranded molecule. This complex formation may result in a range of structural changes to the DNA leading towards the genotoxicity of the drug which can also be exploited in terms of targeted delivery. Here, the insights into the PLM-DNA binding mechanism calls for the further studies related to PLM mode of action related to other biomolecules and to further explore its therapeutic potential, while it gets administered into the human body.

## Data Availability

The original contributions presented in the study are included in the article, further inquiries can be directed to the corresponding authors.

## References

[B1] AhmadA.AhmadM. (2018). Deciphering the mechanism of interaction of edifenphos with calf thymus DNA. Spectrochim. Acta A Mol. Biomol. Spectrosc. 188, 244–251. 10.1016/j.saa.2017.07.014 28732283

[B2] AzizM. H.DreckschmidtN. E.VermaA. K. (2008). Plumbagin, a medicinal plant-derived naphthoquinone, is a novel inhibitor of the growth and invasion of hormone-refractory prostate cancer. Cancer Res. 68, 9024–9032. 10.1158/0008-5472.can-08-2494 18974148PMC2584362

[B3] ChenC. A.ChangH. H.KaoC. Y.TsaiT. H.ChenY. J. (2009). Plumbagin, isolated from Plumbago zeylanica, induces cell death through apoptosis in human pancreatic cancer cells. Pancreatology 9, 797–809. 10.1159/000210028 20110748

[B4] FroehlichE.MandevilleJ. S.WeinertC. M.KreplakL.Tajmir-RiahiH. A. (2011). Bundling and aggregation of DNA by cationic dendrimers. Biomacromolecules 12, 511–517. 10.1021/bm1013102 21192723

[B5] GuanY.ZhouW.YaoX.ZhaoM.LiY. (2006). Determination of nucleic acids based on the fluorescence quenching of Hoechst 33258 at pH 4.5. Anal. Chim. acta 570, 21–28. 10.1016/j.aca.2006.03.106

[B6] HolmA. I. S.NielsenL. M.HoffmannS. V.NielsenS. B. (2010). Vacuum-ultraviolet circular dichroism spectroscopy of DNA: a valuable tool to elucidate topology and electronic coupling in DNA. Phys. Chem. Chem. Phys. 12, 9581–9596. 10.1039/c003446k 20607185

[B7] IvanovV. I.MinchenkovaL. E.SchyolkinaA. K.PoletayevA. I. (1973). Different conformations of double-stranded nucleic acid in solution as revealed by circular dichroism. Biopolymers 12, 89–110. 10.1002/bip.1973.360120109 4687151

[B8] JainS. S.PolakM.HudN. V. (2003). Controlling nucleic acid secondary structure by intercalation: effects of DNA strand length on coralyne-driven duplex disproportionation. Nucleic Acids Res. 31, 4608–4615. 10.1093/nar/gkg648 12888521PMC169941

[B9] KakkarR.GargR.Suruchi (2002). Theoretical study of tautomeric structures and fluorescence spectra of Hoechst 33258. J. Mol. Struct. THEOCHEM 579, 109–113. 10.1016/s0166-1280(01)00721-7

[B10] KumariR.KumarR.LynnA. (2014). g_mmpbsa--a GROMACS tool for high-throughput MM-PBSA calculations. J. Chem. Inf. Model 54, 1951–1962. 10.1021/ci500020m 24850022

[B11] LaiL.LiuJ.ZhaiD.LinQ.HeL.DongY. (2012). Plumbagin inhibits tumour angiogenesis and tumour growth through the Ras signalling pathway following activation of the VEGF receptor-2. Br. J. Pharmacol. 165, 1084–1096. 10.1111/j.1476-5381.2011.01532.x 21658027PMC3346245

[B12] LakowiczJ. R. (2006). Principles of fluorescence spectroscopy. Berlin, Germany: Springer.

[B13] LefstinJ. A.YamamotoK. R. (1998). Allosteric effects of DNA on transcriptional regulators. Nature 392, 885–888. 10.1038/31860 9582068

[B14] LiX. L.HuY. J.WangH.YuB. Q.YueH. L. (2012). Molecular spectroscopy evidence of berberine binding to DNA: Comparative binding and thermodynamic profile of intercalation. Biomacromolecules 13, 873–880. 10.1021/bm2017959 22316074

[B15] LiY.ZhangG.PanJ.ZhangY. (2014). Determination of metolcarb binding to DNA by spectroscopic and chemometrics methods with the use of acridine orange as a probe. Sensors Actuators B Chem. 191, 464–472. 10.1016/j.snb.2013.10.022

[B16] LiuY.CaiY.HeC.ChenM.LiH. (2017). Anticancer properties and pharmaceutical applications of plumbagin: A review. Am. J. Chin. Med. 45, 423–441. 10.1142/s0192415x17500264 28359198

[B17] ManuK. A.ShanmugamM. K.RajendranP.LiF.RamachandranL.HayH. S. (2011). Plumbagin inhibits invasion and migration of breast and gastric cancer cells by downregulating the expression of chemokine receptor CXCR4. Mol. Cancer 10, 107. 10.1186/1476-4598-10-107 21880153PMC3175200

[B18] MergnyJ.Duval-ValentinG.NguyenC.PerrouaultL.FauconB.RougéeM. (1992). Triple helix-specific ligands. Science 256, 1681–1684. 10.1126/science.256.5064.1681 1609278

[B19] NiuM.CaiW.LiuH.ChongY.HuW.GaoS. (2015). Plumbagin inhibits growth of gliomas *in vivo* via suppression of FOXM1 expression. J. Pharmacol. Sci. 128, 131–136. 10.1016/j.jphs.2015.06.005 26154848

[B20] PállS.AbrahamM. J.KutznerC.HessB.LindahlE. (2014). “Tackling exascale software challenges in molecular dynamics simulations with GROMACS,” in Solving Software Challenges for Exascale: International Conference on Exascale Applications and Software, EASC 2014, Stockholm, Sweden, April 2014 (Springer), 3–27.

[B21] RahbanM.DivsalarA.SabouryA. A.GolestaniA. (2010). Nanotoxicity and spectroscopy studies of silver nanoparticle: Calf thymus DNA and K562 as targets. J. Phys. Chem. C 114, 5798–5803. 10.1021/jp910656g

[B22] RajendiranV.MuraliM.SureshE.PalaniandavarM.PeriasamyV. S.AkbarshaM. A. (2008). Non-covalent DNA binding and cytotoxicity of certain mixed-ligand ruthenium(II) complexes of 2,2'-dipyridylamine and diimines. Dalton Trans., 2157–2170. 10.1039/b715077f 18398542

[B23] RamanN.SobhaS.MituL. (2012). Synthesis, structure elucidation, DNA interaction, biological evaluation, and molecular docking of an isatin-derived tyramine bidentate Schiff base and its metal complexes. Monatsh. für Chemie-Chemical Mon. 143, 1019–1030. 10.1007/s00706-011-0699-8

[B24] RehmanS. U.SarwarT.HusainM. A.IshqiH. M.TabishM. (2015). Studying non-covalent drug-DNA interactions. Arch. Biochem. Biophys. 576, 49–60. 10.1016/j.abb.2015.03.024 25951786

[B25] RoyM.BhowmickT.SanthanagopalR.RamakumarS.ChakravartyA. R. (2009). Photo-induced double-strand DNA and site-specific protein cleavage activity of L-histidine (μ-oxo) diiron (III) complexes of heterocyclic bases. Dalton Trans., 4671–4682. 10.1039/b901337g 19513475

[B26] SarkarD.DasP.BasakS.ChattopadhyayN. (2008). Binding interaction of cationic phenazinium dyes with calf thymus DNA: A comparative study. J. Phys. Chem. B 112, 9243–9249. 10.1021/jp801659d 18610959

[B27] SatyanarayanaS.DabrowiakJ. C.ChairesJ. B. (1992). Neither.DELTA.- nor.LAMBDA.-tris(phenanthroline)ruthenium(II) binds to DNA by classical intercalation. Biochemistry 31, 9319–9324. 10.1021/bi00154a001 1390718

[B28] SatyanarayanaS.DabrowiakJ. C.ChairesJ. B. (1993). Tris(phenanthroline)ruthenium(II) enantiomer interactions with DNA: Mode and specificity of binding. Biochemistry 32, 2573–2584. 10.1021/bi00061a015 8448115

[B29] SayedM.KrishnamurthyB.PalH. (2016). Unraveling multiple binding modes of acridine orange to DNA using a multispectroscopic approach. Phys. Chem. Chem. Phys. 18, 24642–24653. 10.1039/c6cp03716j 27545984

[B30] ShahabadiN.FatahiN.MahdaviM.NejadZ. K.PourfouladM. (2011). Multispectroscopic studies of the interaction of calf thymus DNA with the anti-viral drug, valacyclovir. Spectrochimica Acta Part A Mol. Biomol. Spectrosc. 83, 420–424. 10.1016/j.saa.2011.08.056 21930421

[B31] ShahabadiN.HadidiS. (2012). Spectroscopic studies on the interaction of calf thymus DNA with the drug levetiracetam. Spectrochim. Acta A Mol. Biomol. Spectrosc. 96, 278–283. 10.1016/j.saa.2012.05.045 22698844

[B32] ShiJ. H.ChenJ.WangJ.ZhuY. Y. (2015). Binding interaction between sorafenib and calf thymus DNA: Spectroscopic methodology, viscosity measurement and molecular docking. Spectrochim. Acta A Mol. Biomol. Spectrosc. 136, 443–450. 10.1016/j.saa.2014.09.056 25311519

[B33] SinhaS.PalK.ElkhananyA.DuttaS.CaoY.MondalG. (2013). Plumbagin inhibits tumorigenesis and angiogenesis of ovarian cancer cells *in vivo* . Int. J. Cancer 132, 1201–1212. 10.1002/ijc.27724 22806981PMC3496826

[B34] SongY.KangJ.ZhouJ.WangZ.LuX.WangL. (2000). Study on the fluorescence spectra and electrochemical behavior of ZnL2 and Morin with DNA. Spectrochim. Acta A Mol. Biomol. Spectrosc. 56a, 2491–2497. 10.1016/s1386-1425(00)00340-1 11075692

[B35] SubramaniyaB. R.SrinivasanG.SadullahS. S.DavisN.SubhadaraL. B.HalagowderD. (2011). Apoptosis inducing effect of plumbagin on colonic cancer cells depends on expression of COX-2. PLoS One 6, e18695. 10.1371/journal.pone.0018695 21559086PMC3084694

[B36] Uma MaheswariP.PalaniandavarM. (2004). DNA binding and cleavage properties of certain tetrammine ruthenium(II) complexes of modified 1,10-phenanthrolines--effect of hydrogen-bonding on DNA-binding affinity. J. Inorg. Biochem. 98, 219–230. 10.1016/j.jinorgbio.2003.09.003 14729302

[B37] WallaceA. C.LaskowskiR. A.ThorntonJ. M. (1995). Ligplot: A program to generate schematic diagrams of protein-ligand interactions. Protein Eng. 8, 127–134. 10.1093/protein/8.2.127 7630882

[B38] WangG.YanC.WangD.LiD.LuY. (2012). Specific binding of a dihydropyrimidinone derivative with DNA: Spectroscopic, calorimetric and modeling investigations. J. luminescence 132, 1656–1662. 10.1016/j.jlumin.2012.02.021

[B39] WangX.LiY.GongS.FuD. (2002). A spectroscopic study on the DNA binding behavior of the anticancer drug dacarbazine. Spectrosc. Lett. 35, 751–756. 10.1081/sl-120016277

[B40] WijeratneS. S.PatelJ. M.KiangC.-H. (2011). “Melting transitions of DNA-capped gold nanoparticle assemblies,” in Reviews in plasmonics 2010 (Berlin, Germany: Springer), 269–282.

[B41] WilsonW.MizanS.TaniuosF. A.YaoS.ZonG. (1994). The interaction of intercalators and groove-binding agents with DNA triple-helical structures: The influence of ligand structure, DNA backbone modifications and sequence. J. Mol. Recognit. 7, 89–98. 10.1002/jmr.300070206 7826678

[B42] WuH.JiaF.KouF.LiuB.YuanJ.BaiY. (2011). A schiff base ligand N-(2-hydroxylacetophenone)-3-oxapentane-1, 5-diamine and its nickel (II) complex: synthesis, crystal structure, antioxidation, and DNA-binding properties. Transit. Metal. Chem. 36, 847–853. 10.1007/s11243-011-9539-2

[B43] ZhangG.HuX.PanJ. (2011). Spectroscopic studies of the interaction between pirimicarb and calf thymus DNA. Spectrochimica Acta Part A Mol. Biomol. Spectrosc. 78, 687–694. 10.1016/j.saa.2010.11.050 21176886

